The article "Association between Rheumatoid Arthritis Disease Activity and Risk of Ovarian Malignancy in Middle-Aged and Elderly Women" was published in 2022. Journal: Biomed Res Int.

# Association between Rheumatoid Arthritis Disease Activity and Risk of Ovarian Malignancy in Middle-Aged and Elderly Women

**DOI:** 10.1155/2022/1062703

**Published:** 2022-05-25

**Authors:** Zhaowei Huang, Linlin Tan, Yi Ling, Fangqin Huang, Wukai Ma

**Affiliations:** ^1^Graduate School of Guizhou University of Chinese Medicine, Guiyang 52000, China; ^2^Institute of Shanxi Traditional Chinese Medicine, Taiyuan 030000, China; ^3^The Second Affiliated Hospital of Guizhou University of Chinese Medicine, Guiyang 52000, China

## Abstract

**Objective:**

To investigate the risk of ovarian malignancy in middle-aged and elderly women with rheumatoid arthritis (RA) and its correlation with disease activity.

**Methods:**

219 middle-aged and elderly (age ≥ 40) female RA patients who were treated at the Department of Rheumatology and Immunology of the Second Affiliated Hospital of Guizhou University of Traditional Chinese Medicine from August 2019 to September 2020 were selected. Their general information such as age and medical history was collected. RA disease activity-related indicators include rheumatoid factor (RF), anticyclic citrullinated peptide antibody (ACPA), ESR, CRP, and ovarian malignancy risk-related indicators including alpha fetoprotein (AFP), carcinoembryonic antigen (CEA), CA125, CA199, and human epididymis protein 4 (HE4) were detected. According to Risk of Ovarian Malignancy Algorithm (ROMA), they were divided into a low-risk group (ROMA-low, premenopausal: ROMA ≤ 11.4%, postmenopausal: ROMA ≤ 29.9%) and a high-risk group (ROMA-high, premenopausal: ROMA > 11.4%, postmenopausal: ROMA > 29.9%) for ovarian malignancy. Meanwhile, according to the DAS28-ESR, they were divided into the general disease activity group (DAS28-ESR ≤ 5.1) and the high disease activity group (DAS28-ESR > 5.1). SPSS 25.0 software was used to compare the differences among groups and to analyze the correlation between ovarian malignancy risk and RA disease activity.

**Results:**

Compared with the ROMA-low group, the levels of RF, ACCP, CDAI, SDAI, DAS28-ESR, and DAS28-CRP in the ROMA-high group were significantly increased (*P* < 0.05). HE4 and ROMA in the high disease activity group were significantly higher than general disease activity group (*P* < 0.05). Spearman correlation analysis showed that age (*r* = 0.472), RF (*r* = 0.221), ACPA (*r* = 0.156), CDAI (*r* = 0.226), SDAI (*r* = 0.221), DAS28-ESR (*r* = 0.254), DAS28-CRP (*r* = 0.208), medications (*r* = 0.189), and CA199 (*r* = 0.250) were correlated with ROMA (*P* < 0.05). Multivariate regression analysis showed that ESR (OR = 1.11), SDAI (OR = 1.02), DAS28-ESR (OR = 1.33), DAS28-CRP (OR = 1.26), and CA199 (OR = 1.03) were independent risk factors for high risk of ovarian malignancy (*P* < 0.05). Subgroup analysis showed that CA199 is an effect modification factor for DAS28-ESR (*P* < 0.05).

**Conclusion:**

The risk of ovarian malignancy is significantly increased in middle-aged and elderly women with high disease activity with rheumatoid arthritis. In clinical, full attention should be paid to the risk of ovarian malignancy in this population. Screening in time, especially in patients with increased DAS28-ESR and CA199 at the same time, is needed.

## 1. Introduction

Rheumatoid arthritis (RA) is a systemic autoimmune disease. As the disease progresses, it will cause the gradual loss of joint function, which will seriously affect the life and work of patients. The global prevalence rate is about 1%, and women are much higher than men [1]. Studies have found that chronic inflammation caused by RA can induce malignant transformation of cells, and long-existing inflammatory mediators form a microenvironment that promotes cell mutagenesis and activates oncogenes [2]. The abnormal activation and proliferation of T lymphocytes, coupled with the frequent use of immunosuppressive drugs in RA patients, and autoimmune dysfunction affect the immune surveillance function and easily lead to immune escape, all of which increase the risk of tumors in RA patients [2–5]. In long-term clinical practice, we have found that RA patients are prone to increase in CA125 [6, 7], especially in middle-aged and elderly women with high disease activity. CA125 is the most widely used tumor marker for the detection of ovarian cancer. Therefore, it is necessary to assess the risk of ovarian cancer in RA patients and its correlation with disease activity, but there is no research report on the correlation between RA disease activity and ovarian cancer risk. Ovarian cancer is one of the most common malignant tumors in women, and the 5-year survival rate is about 20%-30% [8], but early diagnosis can increase to 89% [9]. In addition to CA125, human epididymis protein 4 (HE4) is a new highly specific ovarian malignant tumor marker and the only indicator for early ovarian cancer screening. Studies have shown that the detection of CA125 combined with HE4 can greatly improve the sensitivity and specificity of early diagnosis of ovarian cancer [9, 10]. Therefore, this study used the risk of ovarian malignancy algorithm (ROMA) associated with HE4 and CA125 levels as the main indicator to explore the risk of ovarian cancer in middle-aged and elderly women with RA and its correlation with disease activity.

## 2. Patients and Methods

### 2.1. Research Population

A total of 219 middle-aged and elderly (age ≥ 40) female RA patients who visited the Rheumatology and Immunology Department of the Second Affiliated Hospital of Guizhou University of Traditional Chinese Medicine from February 2019 to September 2020 were selected. All included RA patients meet the 2010 American Rheumatism Association and the European Union against Rheumatism (ACR/EULAR) RA classification criteria [11]. We exclude patients with other rheumatic immune diseases, tumor history, sex hormone use history, history of ectopic pregnancy, ovariectomy, and history of diagnosis and treatment of serious gynecological diseases. All participants signed an informed consent form, and all procedures performed in the study involving human participants complied with the ethical standards of Guizhou University of Traditional Chinese Medicine and with the 1964 Helsinki Declaration and its later amendments or comparable ethical standards.

### 2.2. Research Methods

The age, height, weight, medical history, tender joints count (TJC), joint swelling count (SJC), patient global assessment (PtGA), physician global assessment (PhGA), glucocorticoids use, and treatment medications were recorded for all subjects. RA disease activity-related indicators and ovarian malignancy risk-related indicators were detected including rheumatoid factor (RF), anticyclic citrullinated peptide antibody (ACPA), ESR, CRP, alpha fetoprotein (AFP), carcinoembryonic antigen (CEA), CA125, CA199, and HE4. Patients were assessed for ovarian malignancy risk and RA disease activity, including ROMA, Clinical Disease Activity Index (CDAI), Simplified Disease Activity Index (SDAI), disease activity score based on ESR and 28 joint counts (DAS28-ESR), and disease activity score based on CRP and 28 joint counts (DAS28-CRP). According to the ROMA, they were divided into a low-risk group (ROMA-low, premenopausal: ROMA ≤ 11.4%, postmenopausal: ROMA ≤ 29.9%) of 138 cases (63%) and a high-risk group (ROMA-high, premenopausal: ROMA > 11.4%, postmenopausal: ROMA > 29.9%) of 81 cases (37%). According to the DAS28-ESR, they were divided into the general disease activity group (DAS28-ESR ≤ 5.1) of 129 cases (58.9%) and high disease activity group (DAS28-ESR > 5.1) of 90 cases (41.1%). We compare the differences between the groups. All laboratory tests were carried out by the Laboratory of the Second Affiliated Hospital of Guizhou University of Traditional Chinese Medicine in strict accordance with the kit instructions. The test methods and catalog numbers and brands of reagents used were listed in the following: ESR (179-2300, Kang Jian Medical) was measured by the Westergren method. RF (998-40391, FUJIFILM Wako Pure Chemical Corporation) and CRP (994-65391, FUJIFILM Wako Pure Chemical Corporation) were measured by immunoturbidimetry. ACPA (5031656190, Roche), HE4 (5950929190, Roche), AFP (33210, Beckman Coulter), CEA (33200, Beckman Coulter), CA199 (387687, Beckman Coulter), and CA125 (386357, Beckman Coulter) were measured by chemiluminescence.

### 2.3. Clinical Status and Biochemical Assessment

According to the disease-modifying antirheumatic drugs (DMARDs) used, they were divided into three groups, the csDMARDs group (use conventional synthetic DMARDs only), the tsDMARDs group (use targeted synthetic DMARDs only or in combination), and the bDMARDs group (use biologic DMARDs only or in combination). csDMARDs include methotrexate (MTX), hydroxychloroquine, leflunomide, and sulfasalazine. tsDMARDs include JAK inhibitors (tofacitinib, baricitinib). bDMARDs include TNF inhibitors (etanercept, adalimumab, infliximab, and golimumab) and IL-6 receptor inhibitors (tocilizumab). Glucocorticoid use was divided into two situations: whether there is long-term (≥3 months) use of glucocorticoids or not. Multiple methods were used for assessing disease activity in RA patients. Formula for CDAI is as follows: CDAI = TJC + SJC + PtGA + PhGA. Formula for SDAI is as follows: SDAI = TJC + SJC + PtGA + PhGA + CRP; the unit of CRP is mg·dL^−1^. Formula for DAS28-ESR is as follows: DAS28‐ESR = [0.56 × sqrt(TJC) + 0.28 × sqrt(SJC) + 0.7 × LN(ESR)] × 1.08 + 0.16, sqrt means square root and the unit of ESR is mm·h^−1^. DAS28-ESR ≤ 5.1 into the general disease activity group. DAS28-ESR > 5.1 into the high disease activity group. Formula for DAS28-CRP is as follows: DAS28‐CRP = [0.56 × sqrt(TJC) + 0.28 × sqrt(SJC) + 0.36 × LN(CRP + 1)] × 1.10 + 1.15, where sqrt means square root and the unit of CRP is mg·L^−1^. Ovarian malignancy risk assessment uses the ROMA index. Formula for ROMA is as follows: Premenopausal Prediction Index (PI) = −12.0 + 2.38 × LN(HE4) + 0.0626 × LN(CA125), Postmenopausal Predictive Index (PI) = −8.09 + 1.04 × LN(HE4) + 0.732 × LN(CA125), and ROMA = exp(PI)/[1 + exp(PI)] × 100, where exp represents the *n*th power with *e* as the base, the unit of HE4 is pmol·L^−1^ and the unit of CA125 is U·mL^−1^. According to the reference standards provided by the kit instructions and literature [12], CA125 > 35 U·mL^−1^ is positive (CA125+). CA125 ≤ 35 U·mL^−1^ is negative (CA125-). For premenopausal women, HE4 > 68.96 pmol·L^−1^ is positive (HE4+). ROMA > 11.4% means high risk of ovarian malignancy, and ROMA ≤ 11.4% means low risk. For postmenopausal women, the critical values of HE4 and ROMA are 114.9 pmol·L^−1^ and 29.9%.

### 2.4. Statistical Analysis

Statistical analyses were performed using *SPSS25.0*. Continuous variables with a normal distribution and homogeneity of variance are represented by ($\bar{X}\pm S$), and comparisons between groups are performed by *t*-test. Continuous variables that do not conform to the normal distribution are represented by the median (interquartile range) (M (P25-P75)) and comparisons between groups are performed by the Mann–Whitney *U* test. Categorical variables are expressed in terms of quantity and percentage (*n*, %), and the *χ*^2^ test is used. For the correlation analysis between two variables, the Pearson correlation coefficient is used for the normally distributed variables and the Spearman correlation coefficient is used for the nonnormal variables. Multivariate regression analysis was performed for possible risk factor variables adjusting for confounding variables. Subgroup analyses were performed for the independent risk factors for ovarian malignancy with the largest relative risk. The above test methods were all statistically significant with *P* < 0.05.

## 3. Results

### 3.1. Clinical Status and Biochemical Outcomes

219 patients were included in this study, the age was 60 ± 11.8 years, the median disease duration was 93 months, the median DAS28-ESR was 4.74, 206 patients (94.1%) were without long-term glucocorticoids, the median ROMA risk index was 20.6%, and 81 patients (37%) were at high risk of ovarian cancer malignancy (for more, see Table 1).

### 3.2. Comparison between Groups

Grouped by ROMA index. 138 cases (63%) were at low risk of ovarian malignancy and 81 cases (37%) were at high risk of ovarian malignancy. Compared with the ROMA-low group, RF, ACPA, CDAI, SDAI, DAS28-ESR, and DAS28-CRP in the ROMA-high group were significantly increased (*P* < 0.05). Compared with the csDMARDs group, the high-risk ratio of ovarian malignancy in the bDMARDs group was significantly increased (*P* < 0.05), (see Table 2). Grouped by DAS28-ESR, there were 129 cases (58.9%) in the moderate-low disease activity group and 90 cases (41.1%) in the high disease activity group. Compared with the moderate-low disease activity group, the high disease activity group had significantly higher HE4, ROMA index, and the high-risk ratio of ovarian malignancy (*P* < 0.05), (see Table 3).

### 3.3. Correlation Analysis of ROMA

Correlation analysis showed that age (*r* = 0.472), RF (*r* = 0.221), ACPA (*r* = 0.156), ESR (*r* = 0.272), CRP (*r* = 0.174), CDAI (*r* = 0.226), SDAI (*r* = 0.221), DAS28-ESR (*r* = 0.254), DAS28-CRP (*r* = 0.208), medications (*r* = 0.189), and CA199 (*r* = 0.250) were correlated with ROMA index (*P* < 0.05), (see Table 4).

### 3.4. Regression Analysis of ROMA-High

Factors that may increase ROMA-high were included in the regression equation but avoid including variables that influence each other together. Multivariate regression analysis after adjusting for confounding variables showed that ESR (OR = 1.11), SDAI (OR = 1.02), DAS28-ESR (OR = 1.33), DAS28-CRP (OR = 1.26), and CA199 (OR = 1.03) were independent risk factors for high risk of ovarian malignancy (*P* < 0.05), (see Table 5).

### 3.5. Subgroup Analysis of DAS28-ESR

Commonly used cut-off points in the clinical lead to uneven grouping and reduced statistical performance, so the median of variables that may interact with DAS28-ESR was used as the cut-off point to divide patients into two subgroups. Multivariate analysis showed that total (OR = 1.33), CA199 < 9.69 group (OR = 0.94), and CA199 ≥ 9.69 group (OR = 2.00). There is an interaction between DAS28-ESR and CA199. CA199 is an effect modification factor for DAS28-ESR (*P* < 0.05) (see Table 6).

## 4. Discussion

Long-term immune dysregulation associated with RA development and the resulting chronic inflammation lead to an increased risk of cancer development. Simon et al. [13] performed a meta-analysis about the risk of overall malignancy. This data suggested that patients with RA have an overall increased risk of developing cancer by 10% over the general population. Much evidence suggests that patients with RA have a significantly increased risk of lymphoma and lung cancer [14–20]. Lymphoma may be associated with MTX and bDMARDs in RA patients [14–16]. And it was found that the higher the disease activity, the higher the relative risk [18], which is similar to the conclusion of our study. The latest clinical trial on ovarian cancer risk in RA patients comes from Japan. Inose et al. [21] found MTX and bDMARDs were significantly associated with ovarian cancer. In addition, concomitant use of bDMARDs further increased the risk of breast, ovarian, and lung cancers in MTX-treated patients with rheumatoid arthritis. This is similar to the regression analysis results of our study. Świerkot et al. [22] also showed that RA patients with rheumatoid arthritis have an increased risk of cancer, including ovarian cancer. MicroRNA-223 (miR-223) expression is upregulated in rheumatoid arthritis and ovarian cancer tissues [23]. miR-223 can promote ovarian cancer cell proliferation, migration, and invasion in vitro, and promoted tumor growth in vivo. All of the above evidence points to an increased risk of ovarian cancer in RA patients.

The mortality rate of ovarian cancer ranks first in the world for female reproductive system tumors, and the main reason is that it is difficult to diagnose early. CA125 is a mucin-type glycoprotein associated with ovarian cancer. It is produced by the MUC16 gene and is the most widely used tumor marker for clinical detection of ovarian cancer. It first appeared in the 1980s, and Bast et al. [24]. isolated OC125 monoclonal antibody specifically in cancerous ovarian tissue. The vast majority of patients with ovarian cancer have elevated CA125 at least 4 months before diagnosis [25]. In the clinic, we found that RA patients often have an abnormal increase in CA125 [26], especially middle-aged and elderly women in the active stage of the disease. Our research has also confirmed this. This inspires us to think, will this population increase the risk of ovarian cancer? However, the CA125 test alone has low specificity for the diagnosis of ovarian cancer. Serum CA125 levels may also increase in physiological or pathological conditions such as menstruation, pregnancy, peritoneal inflammation, and endometriosis [27]. False positives are prone to occur, so we need more suitable biomarkers for the diagnosis of ovarian tumors. HE4 is a breakthrough in the diagnosis of ovarian cancer in the 21st century. The specificity of ovarian cancer diagnosis can reach 90%. It is only highly expressed in ovarian cancer and is low in benign tumors and endometriosis [28–30]. Other studies have also confirmed that the gene encoding HE4 is not overexpressed in endometriotic lesions [31]. Our research results found that among RA patients, patients with high disease activity have higher HE4 levels and positive rates than those with low disease activity. This means that high disease activity will increase the risk of ovarian cancer, and the results of ROMA also reflect this. ROMA is a risk of ovarian malignancy algorithm first proposed by Moore and McMeekin in 2009 [32]. It is a regression model that correlates HE4 and CA125 levels according to menopausal status. Studies have shown that when the two markers of HE4 and CA125 are used together, the sensitivity and specificity of predicting ovarian malignant tumors are significantly improved [33–36], which can greatly reduce the false positive rate of CA125. A study by Ortiz-Muñoz et al. [37] proved that ROMA can help stratify patients with unclear clinical diagnoses. The study showed that the sensitivity of ROMA to distinguish ovarian cancer from benign gynecological diseases was 93.1%, the specificity was 90.7%, the positive predictive value (PPV) was 98.2%, and the negative predictive value (NPV) was 71.1%. An Italian multicenter study involving 387 participants also believes that ROMA has the best diagnostic performance in the early diagnosis of ovarian cancer [38]. Our research shows that patients' ROMA is positively correlated with RA disease activity indicators. Compared with the ovarian malignancy low-risk group, the high-risk group had significantly higher RF, ACCP, CDAI, SDAI, DAS28-ESR, and DAS28-CRP levels. This suggests that high disease activity in RA is associated with a high risk of ovarian malignancy.

RA is a chronic inflammatory autoimmune disease. Studies have shown that patients with rheumatoid arthritis have an increased risk of cancer [2–5, 39]. The long-term chronic inflammatory microenvironment, the secretion of immunosuppressive factors such as IL-10, abnormal autoimmune response, and the use of immunosuppressive drugs have led to frequent tumor-like symptoms and paraneoplastic syndromes in RA patients. This may be because prolonged immunosuppression may affect the immune surveillance function of the immune system and cause the immune escape of tumor cells. Therefore, it is very important to assess the risk of cancer in RA patients. Multijoint immune inflammation is the main manifestation of RA. ESR and CRP are common indicators of inflammation in clinical practice. RF and ACPA are important serological criteria for the diagnosis of RA. Their persistent high titer positivity is a preliminary reflect the activity of RA to some extent, although sometimes not completely accurate. RF and ACPA were statistically different in group comparisons, but not in multivariate analysis after adjusting for confounding variables, probably because they correlated with disease activity. The 28 joint count disease activity score (DAS28), CDAI, and SDAI are the most commonly used clinical indexes to evaluate RA disease activity. It combines the tender joints count, the joint swelling count, patient global assessment, physician global assessment, and inflammation indicators. It can accurately and comprehensively assess the disease activity degree of RA patients. Our findings found that RF and bDMARDs were statistically significant on univariate analysis but not after adjustment for confounding variables. Therefore, there may be a correlation between RF, bDMARDs, and ROMA index, but more experiments are needed to confirm. Multivariate analysis showed ESR, SDAI, DAS28-ESR, DAS28-CRP, and CA199 are all independent risk factors for increased ovarian malignancy risk in middle-aged and elderly women with RA. DAS28-ESR had the largest odds ratio, so we further performed a subgroup analysis on DAS28-ESR. The interaction between DAS28-ESR and CA199 was found. CA199 is a serum marker of ovarian cancer. The data from Lertkhachonsuk et al. [40] showed that elevated CA199 was an independent risk factor for ovarian tumors (OR = 1.74, 95% CI = 1.22-2.47) and was a better predictor. This is consistent with our findings. In addition, CA199 combined with other tumor markers can improve the sensitivity and specificity of ovarian cancer diagnosis [41]. And CA199 level is correlated with the survival of ovarian cancer patients [42]. It is clear that RA patients with high disease activity and high CA199 levels have a higher risk of ovarian cancer.

This study was inspired by the abnormal increase of CA125 in middle-aged and elderly women with RA. For the first time, the disease activity of RA patients was correlated with the risk of ovarian malignancy algorithm. Our study found that middle-aged and older women with rheumatoid arthritis with high disease activity had a significantly increased risk of ovarian malignancy. Among them, the patients with high disease activity and high CA199 levels are a special population with an extremely high risk of ovarian malignancy. The limitation of the study is that it is only a preliminary exploratory study. Long-term follow-up results are needed to compare the actual incidence of ovarian cancer in RA populations with different disease activities. Guizhou Province is located in the remote and relatively backward southwest region of China. Patients have poor health consciousness, and many RA patients develop joint deformities before they come to see a doctor. Diagnosis and the actual course of disease are very different. Therefore, the results related to the course of the disease are open to debate. Finally, the study is a cross-sectional study, which can only show that there is a close relationship between disease activity and the risk of ovarian malignancy in RA patients but cannot clarify the causal relationship between the two.

## 5. Conclusion

Middle-aged and elderly women with rheumatoid arthritis with high disease activity have a significantly increased risk of ovarian malignancy. In clinical practice, full attention should be paid to the risk of ovarian cancer in this population, and timely investigation should be carried out, especially in patients with increased DAS28-ESR and CA199 at the same time.

## Figures and Tables

**Table 1:** Clinical status and biochemical outcomes.

Variables	RA (*n* = 219)
Age (years)	60.4 ± 11.9
BMI (kg·m^−2^)	22.1 ± 3.0
Disease duration (months)	93 (19-139)
RF (U·L^−1^)	88.5 (33.1-190.9)
ACPA	105.6 (14.9-400)
ESR (mm·h^−1^)	41 (21-73)
CRP (mg·L^−1^)	10.6 (3.0-35.3)
TJC (*n*)	5 (2-10)
SJC (*n*)	2 (1-6)
CDAI	18 (12-29)
SDAI	19.8 (12.5-33)
DAS28-ESR	4.74 (3.45-5.92)
DAS28-CRP	3.90 (2.66-5.24)
Long-term (≥3 months)glucocorticoids	
No	206 (94.1)
Yes	13 (5.9)
Medications	
csDMARDs	131 (59.8)
tsDMARDs	38 (17.4)
bDMARDs	50 (22.8)
CA125 (U·mL^−1^)	17.1 (12.3-25.9)
CA125+, *n* (%)	25 (11.4)
HE4 (pmol·L^−1^)	86.3 (63.1-131.5)
HE4+, *n* (%)	82 (37.4)
ROMA (%)	20.6 (13.3-32.5)
ROMA-high, *n* (%)	81 (37)
AFP (ng·mL^−1^)	2.66 (1.89-3.7)
CEA (ng·mL^−1^)	1.89 (1.21-3.06)
CA199 (U·mL^−1^)	9.69 (6.36-15.47)

**Table 2:** Comparison between the ROMA-low group and ROMA-high group.

Variables	ROMA-low(*n* = 138)	ROMA-high(*n* = 81)	*P* value
Age (years)	59.5 ± 10.8	61.9 ± 13.4	0.168
BMI (kg·m^−2^)	22.2 ± 3.0	22.0 ± 3.2	0.589
Disease duration (months)	93.5 (17.5-141.3)	92.0 (24.5-135)	0.874
RF (U·L^−1^)	62.9(24.6-155.1)	141(72-204.3)	<0.001^∗^
ACPA (RU·mL^−1^)	68.2 (10.5-400)	150.5 (38.0-400)	0.027^∗^
ESR (mm·h^−1^)	35.0 (16.0-69.3)	54.0 (28.5-76.5)	0.001^∗^
CRP (mg·L^−1^)	8.6 (2.0-32.1)	20.0 (5.1-44.1)	0.004^∗^
CDAI	17 (9.8-26.3)	21 (15-32.5)	0.002^∗^
SDAI	17.9 (10-29)	21.9 (15.5-36.1)	0.002^∗^
DAS28-ESR	4.5 (3.08-5.51)	5.18 (4.2-6.27)	0.001^∗^
DAS28-CRP	3.59 (2.31-4.89)	4.31 (3.19-5.45)	0.002^∗^
Long-term (≥3 months)glucocorticoids			
No	131 (94.9)	75 (92.6)	0.480
Yes	7 (5.1)	6 (7.4)	
Medications			
csDMARDs	89 (64.5)	42 (51.9)	Reference
tsDMARDs	23 (16.7)	15 (18.5)	0.395
bDMARDs	26 (18.8)	24 (29.6)	0.046^∗^
CA125 (U·mL^−1^)	14.5 (11-19.4)	25.8 (18.9-34.4)	<0.001^∗^
HE4 (pmol·L^−1^)	70.1 (57.5-94.3)	141.8 (103.7-195)	<0.001^∗^
ROMA (%)	16.2 (11.3-21.6)	37.4 (30.8-45.3)	<0.001^∗^
AFP (ng·mL^−1^)	2.65 (1.98-3.97)	2.73 (1.83-3.44)	0.637
CEA (ng·mL^−1^)	2.03 (1.24-3.41)	1.64 (1.17-2.67)	0.049^∗^
CA199 (U·mL^−1^)	9.3 (6.27-14.23)	10.16 (6.73-17.3)	0.169

Note: ^∗^A significant difference (*P* < 0.05) between two groups.

**Table 3:** Comparison between the general disease activity group and high disease activity group.

Variables	DAS28-ESR ≤ 5.1(*n* = 129)	DAS28-ESR > 5.1(*n* = 90)	*P* value
Age (years)	60.5 ± 12.1	60.2 ± 11.6	0.813
BMI (kg·m^−2^)	22.3 ± 3.1	21.8 ± 3.0	0.287
Disease duration (months)	91.0 (8.5-134.5)	96.5 (29-150.8)	0.076
RF (U·L^−1^)	61.6 (24.3-140.7)	144.9 (70.9-201.8)	<0.001^∗^
ACPA (RU·mL^−1^)	62.9 (11.1-400)	190.4 (33.5-400)	0.002^∗^
CDAI	13 (9-17)	31 (25-40)	<0.001^∗^
SDAI	13.2 (9.2-18.3)	35.2 (27.1-46.6)	<0.001^∗^
DAS28-ESR	3.71 (2.88-4.51)	6.18 (5.50-6.72)	<0.001^∗^
DAS28-CRP	2.97 (2.19-3.68)	5.45 (4.77-6.15)	<0.001^∗^
Long-term (≥3 months)glucocorticoids			
No	124 (96.1)	82 (91.1)	0.122
Yes	5 (3.9)	8 (8.9)	
Medications			
csDMARDs	88 (68.2)	43 (47.8)	Reference
tsDMARDs	18 (14.0)	20 (22.2)	0.026^∗^
bDMARDs	23 (17.8)	27 (30)	0.009^∗^
CA125 (U·mL^−1^)	17.2 (12.7-25.0)	16.7 (12-27.5)	0.616
CA125+, *n* (%)	12 (9.3)	13 (14.4)	0.239
HE4 (pmol·L^−1^)	79.1 (61.6-116.4)	96.6 (66.7-147.9)	0.007^∗^
HE4+, *n* (%)	40 (31.0)	42 (46.7)	0.018^∗^
ROMA (%)	18.6 (12.6-29.1)	24.5 (14.1-37.7)	0.026^∗^
ROMA-high, *n* (%)	40 (31.0)	41 (45.6)	0.028^∗^
AFP (ng·mL^−1^)	2.68 (1.98-3.85)	2.64 (1.84-3.65)	0.687
CEA (ng·mL^−1^)	1.97 (1.19-2.86)	1.87 (1.24-3.15)	0.998
CA199 (U·mL^−1^)	9.98 (6.18-17.00)	9.47 (6.78-13.48)	0.469

^∗^A significant difference (*P* < 0.05) between two groups.

**Table 4:** Correlation analysis of ROMA.

Variables	ROMA	
	*r*	*P* value
Age	0.472	<0.001^∗^
BMI	-0.054	0.429
Disease duration	0.025	0.714
RF	0.221	0.001^∗^
ACPA	0.156	0.021^∗^
ESR	0.272	<0.001^∗^
CRP	0.174	0.01^∗^
CDAI	0.226	0.001^∗^
SDAI	0.221	0.001^∗^
DAS28-ESR	0.254	<0.001^∗^
DAS28-CRP	0.208	0.002^∗^
Long-termglucocorticoids	0.049	0.467
Medications	0.189	0.005^∗^
AFP	-0.082	0.227
CEA	-0.123	0.069
CA199	0.250	<0.001^∗^

Note: ^∗^Statistically significant correlations (*P* < 0.05).

**Table 5:** Regression analysis of ROMA-high.

Variables	ROMA-high (univariate)		ROMA-high (multivariate)	
	OR (95% CI)	*P*	OR (95% CI)	*P*
Age (years)	1.02 (0.994-1.041)	0.145	1.01 (0.986-1.039)	0.363
Disease duration (months)	1.00 (0.997-1.004)	0.881	1.00 (0.994-1.003)	0.511
RF (U·dL^−1^)	1.05 (1.017-1.087)	0.003^∗^	1.04 (0.997-1.075)	0.072
ACPA (RU·mL^−1^)	1.00 (1.000-1.003)	0.172	1.00 (0.999-1.002)	0.408
ESR (cm·h^−1^)	1.13 (1.040-1.235)	0.004^∗^	1.11 (1.012-1.225)	0.027^∗^
CRP (mg·dL^−1^)	1.10 (1.022-1.182)	0.011^∗^	1.07 (0.997-1.158)	0.059
CDAI	1.04 (1.011-1.059)	0.004^∗^	1.03 (0.999-1.052)	0.059
SDAI	1.03 (1.009-1.045)	0.003^∗^	1.02 (1.000-1.040)	0.048^∗^
DAS28-ESR	1.42 (1.167-1.722)	<0.001^∗^	1.33 (1.070-1.652)	0.010^∗^
DAS28-CRP	1.34 (1.118-1.609)	0.002^∗^	1.26 (1.028-1.536)	0.026^∗^
Long-term (≥3 months)glucocorticoids				
No	Reference	/	Reference	/
Yes	1.50 (0.485-4.620)	0.483	0.87 (0.232-3.259)	0.831
Medications				
csDMARDs	Reference	/	Reference	/
tsDMARDs	1.38 (0.655-2.916)	0.396	1.13 (0.494-2.583)	0.773
bDMARDs	1.96 (1.006-3.804)	0.048^∗^	1.56 (0.738-3.291)	0.244
AFP (ng·mL^−1^)	0.91 (0.758-1.085)	0.285	0.96 (0.787-1.179)	0.716
CEA (ng·mL^−1^)	0.78 (0.637-0.956)	0.017^∗^	0.81 (0.650-1.013)	0.064
CA199 (U·mL^−1^)	1.02 (1.002-1.047)	0.036^∗^	1.03 (1.001-1.049)	0.043^∗^

Note: ^∗^Statistically significant (*P* < 0.05).

**Table 6:** Subgroup analysis of DAS28-ESR.

Group	*n* (%)	DAS28-ESR	Crude		*P* for interaction	Adjusted		*P* for interaction
			OR (95% CI)	*P* value		OR (95% CI)	*P* value	
Total	219	4.74 (3.45-5.92)	1.42 (1.167-1.722)	<0.001^∗^	/	1.33 (1.070-1.652)	0.010^∗^	/
Age (years)								
Age < 60	108 (49)	4.61 (3.41-5.92)	1.34 (1.014-1.769)	0.040^∗^	0.638	1.52 (1.049-2.189)	0.027^∗^	0.879
Age ≥ 60	111 (51)	4.77 (3.50-5.95)	1.50 (1.135-1.974)	0.004^∗^		1.26 (0.900-1.762)	0.178	
RF (U·L^−1^)								
RF < 89	109 (50)	4.26 (3.09-5.25)	1.35 (0.996-1.841)	0.053	0.074	1.18 (0.803-1.725)	0.404	0.051
RF ≥ 89	110 (50)	5.29 (3.92-6.30)	1.30 (0.997-1.705)	0.053		1.35 (1.003-1.807)	0.047^∗^	
ACPA (RU·mL^−1^)								
ACPA < 105.6	109 (50)	4.11 (2.98-5.34)	1.45 (1.096-1.924)	0.009^∗^	0.123	1.25 (0.908-1.717)	0.172	0.251
ACPA ≥ 105.6	110 (50)	5.14 (4.20-6.30)	1.30 (0.978-1.736)	0.071		1.49 (1.060-2.083)	0.021^∗^	
AFP (ng·mL-1)								
AFP < 2.66	109 (50)	4.82 (3.54-6.06)	1.40 (1.067-1.840)	0.015^∗^	0.736	1.40 (1.007-1.957)	0.172	0.661
AFP ≥ 2.66	110 (50)	4.61 (3.38-5.80)	1.44 (1.091-1.911)	0.010^∗^		1.29 (0.911-1.831)	0.150	
CEA (ng·mL-1)								
CEA < 1.89	108 (49)	4.77 (3.63-6.14)	1.33 (1.021-1.719)	0.034^∗^	0.951	1.26 (0.931-1.697)	0.136	0.598
CEA ≥ 1.89	111 (51)	4.69 (3.28-5.70)	1.53 (1.135-2.005)	0.005^∗^		1.56 (1.086-2.247)	0.016^∗^	
CA199 (U·mL^−1^)								
CA199 < 9.69	108 (49)	4.87 (3.38-6.21)	1.10 (0.849-1.432)	0.462	0.014^∗^	0.94 (0.676-1.293)	0.685	0.010^∗^
CA199 ≥ 9.69	111 (51)	4.58 (3.49-5.70)	2.05 (1.467-2.871)	<0.001^∗^		2.00 (1.387-2.880)	<0.001^∗^	

Note: ^∗^Statistically significant (*P* < 0.05).

## Data Availability

The data used to support the findings of this study are available from the corresponding author upon request.
